The article "Redactable Blockchain Trust Scheme Based on Reputation Consensus for MEC" was published in 2022. Journal: Comput Intell Neurosci.

# Redactable Blockchain Trust Scheme Based on Reputation Consensus for MEC

**DOI:** 10.1155/2022/3269445

**Published:** 2022-04-28

**Authors:** YongLi Tang, Shuai Wu, XiaoJun Wang

**Affiliations:** ^1^School of Computer Science and Technology, Henan Polytechnic University, Jiaozuo 454003, China; ^2^School of Electronic Engineering, Dublin City University, Dublin 9, Ireland

## Abstract

Blockchain technology can build trust, reduce costs, and accelerate transactions in the mobile edge computing (MEC) and manage computing resources using the smart contract. However, the immutability of blockchain also poses challenges for the MEC, such as the smart contract with bugs cannot be modified or deleted. We propose a redactable blockchain trust scheme based on reputation consensus and a one-way trapdoor function in response to the problem that data on the blockchain, which is an error or invalid needs to be modified or deleted. The scheme calculates each user's reputation based on their currency age and behavior. The SM2 asymmetric cryptography algorithm is used as the one-way trapdoor function to construct a new Merkle tree structure, which guarantees the legitimacy of the modification or deletion after verification and vote. The simulation experiments show that the modification or deletion does not change the existing blockchain structure and the links of blocks. Furthermore, the consensus verification accurately passes after the modification or deletion operations, which indicates the proposed scheme is feasible.

## 1. Introduction

The mobile edge computing (MEC) reduces latency and network load by consolidating computing resources that are close to mobile users in edge networks. However, there are problems in system security and resource management. The security and privacy of MEC have been a concern in recent years, and blockchain can provide the best solution. Blockchain technology is one of the revolutionary emerging technologies in recent years. The immutability of blockchain technology facilitates it to establish a consensus in a trustless environment [1]. Furthermore, blockchain has the advantages of decentralization, detrust, anonymity, and data incorruptibility, and makes the transmission of secret information in the MEC more secure [2]. Therefore, it has broad development prospects. The smart contract can realize the decentralized resource management and ensure the security of system data. Using the decentralized characteristics of blockchain to perform task allocation and scheduling in mobile edge computing can effectively eliminate the attack behavior to the central server and ensure the correctness of data transmission.

Blockchain brings benefits to the MEC but also challenges. The immutability ensures the information security of the computing devices on the chain. It also means the wrong or invalid information cannot be modified or deleted and will be permanently stored in the blockchain. The smart contract can facilitate the intelligent management of MEC devices. Still, bugs in the smart contract will lead to irreparable damage, as in the well-known DAO attack. However, illegal information has been maliciously uploaded to the blockchain time and again since the creation of blockchain, providing opportunities for criminals to disrupt the order of the blockchain network for benefit. The current research and application of blockchain emphasize the security of storage and transmission of data on the blockchain, while ignoring the security of data contained on the blockchain from the perspective of information regulation [3]. Data on the blockchain can only be appended, not deleted or modified [4]; the storage burden of the entire blockchain increases due to the increasing amount of data on the blockchain, which cannot be deleted or altered, which is not conducive to maintaining. The General Data Protection Regulation (GDPR) mandated by the European Union in 2018 sets new standards for collecting, storing, protecting, and using users' data. Companies need to ask for each user's permission before collecting their personal data. The user has the right to be forgotten, and the data controllers must ensure that personal data are accurate and kept up to date. It means that users can withdraw their permission at any time and ask companies to modify or delete their personal data. Therefore, the blockchain system applied in this context must provide users with a convenient way to modify or delete. The decentralization of blockchain does not mean that the system data cannot be modified, but the data on the blockchain can be modified with the approval of the majority of the system users, and the modification operation is performed by the system users, which does not violate the concept of decentralization. Therefore, the study of redactable blockchain technology under specific conditions is of great research significance.

After Satoshi Nakamoto proposed “Bitcoin: A Peer-to-Peer Electronic Cash System” in 2008 [5], blockchain came into the public eye. As the core technology of blockchain, the consensus mechanism determines blockchain's security, scalability, decentralization, and other essential characteristics [6]. It solves the Byzantine problem so that communication between untrustworthy nodes is possible and makes the distributed data of blockchain consistent. A suitable consensus mechanism improves the performance and efficiency of a blockchain system, provides a robust security guarantee, and supports complex application scenarios [7]. The initial Bitcoin blockchain used the Proof-of-Work (PoW) mechanism, which relies highly on the HashRate of nodes, to ensure the consistency of the distributed data. However, PoW proved to be a severe waste of resources and an inefficient transaction. The Proof-of-Stake (PoS) consensus created by Peercoin solves the problem of waste of resources of PoW. However, it cannot resist the permanent divergence. It may lead to polarization, widening the gap between rich and poor nodes, and a low level of decentralization is detrimental to currency circulation [8]. Liu proposed a new consensus mechanism based on reputation in 2019 (Proof of Reputation, PoR) [9]. It distributes a reputation value to each node and determines who has the right to create a new block according to the reputation value. The PoR consensus mechanism does not waste the HashRate or power resources; it has a low computational cost and is more efficient compared with the PoW consensus mechanism. The PoR also does not lead to polarization compared with the PoS consensus mechanism. The reputation value is logarithmically proportional to the amount of currency. The reputation value increases with the increasing amount of currency, but the growth rate decreases. It allows moderately wealthy nodes to create a new block for rewards.

Krawczyk H proposed the chameleon hash function in 2000 [10], which has a trapdoor that can construct a hash collision. The Accenture company applied for a patent of redactable blockchain that having a trapdoor can modify the block data without changing the block's hash value. Still, the scheme is not secure because the trapdoor is controlled by only one party, and the scheme is highly centralized. Li proposed a study of redactable blockchain technology based on chameleon hash functions and verifiable secret sharing in 2018 [11]. Li's scheme solves the problem of high centralization, with N nodes cooperating to perform modification operations. Still, most of the blockchains are mainly based on traditional collision-resistant hash functions, so the application value of Li's scheme is low. Ren proposed a redactable blockchain scheme based on Proof-of-Space consensus and collision-resistant hash functions in 2020 [12], using one-way trapdoor functions to modify the data on the blockchain. The blockchain structure of Proof of Space is different from Proof of Work and Proof of Stake, due to the features of Proof-of-Space consensus, and this scheme [13] is only limited to Proof-of-Space consensus, which has substantial limitations; the modification involves the inverse operation of Q users. The more users there are in the blockchain network, the larger the Q is, and the lower the efficiency is. Therefore, the Proof of Reputation has many advantages compared with Proof of Space. First, the Proof of Reputation selects a Leader to create a new block according to user's reputation value, and it does not waste the HashRate resources compared with Proof of Space; second, the efficiency of Proof of Space will decrease with the increasing number of Q users in the network, there are Q inverse operations, and the efficiency of Proof of Reputation will not decrease because there is only one inverse operation.

This paper uses a collision-resistant hash function to implement a redactable blockchain scheme based on the Proof of Reputation consensus mechanism (PoR). We propose a new Merkle tree structure using a one-way trapdoor function. As a result, legitimate modification of invalid or error information could be performed after verification without changing the existing blockchain structure; all users can verify the validity of modified data [14].

## 2. Basic Knowledge

### 2.1. One-Way Trapdoor Function

A one-way trapdoor function contains two features: a one-way function and a trapdoor. The one-way function is irreversible. For a one-way function *y* = *f*(*x*), it is easy to calculate *y* given *x* but is computationally infeasible to compute *x* given *y*. There exists a *z* such that we can easily calculate *x* = *f* ^−1^(*y*) if we have *z* and *y*. The function *y* = *f*(*x*) is called one-way trapdoor function, and *z* is called the trapdoor. The character of the one-way function determines its computational complexity, and the character of the trapdoor determines that *z* will be the key to cracking the one-way function.

### 2.2. PoR Consensus-Based Blockchain

A new consensus mechanism based on Proof of Reputation (PoR) was proposed in [9]. The PoR consensus mechanism has certain merits in energy-saving and computation efficiency compared with PoW. Furthermore, PoR can avoid the waste of resources caused by PoW and create a secure network atmosphere.

As shown in Figure 1 [9], the block structure of the PoR consensus mechanism has three parts: block header, transaction sub-block, and reputation sub-block. Detailed contents of the three parts are as follows:

1. Block header: contains block height, version, timestamp, signature of the block header, hash of the previous block (only hash the block header), transaction Merkle root, and reputation Merkle root.
2. Transaction sub-block: contains transactions stored as a Merkle tree. The root of Merkle tree in the transaction sub-block links to the transaction Merkle root in the block header.
3. Reputation sub-block: contains the vote information. As shown in Figure 2, the vote information includes explicitly: the voter's public key, reputation value, opinion of agreement or disagreement, signature, and the block hash. The vote information, stored as a Merkle tree, is used to verify the legitimacy of the created block. The Merkle root links to the reputation Merkle root in the block header.

In the PoR consensus mechanism, the highest reputation node can create a new block. The factors that affect a node's reputation are as follows: currency age *R*_*s*_; transaction activities with other nodes *R*_*a*_; and contribution to consensus *R*_*c*_. The currency age is the product of currency amount and time; transactions with other honest nodes and participation in consensus validation voting will increase a node's reputation value, and the reputation values of each participating node will change when each block is published, whether the block is approved or rejected by the network. The following equations computing the constituting components, *R*_*s*_, *R*_*a*_, and *R*_*c*_, of the reputation values are formulated in [9].

(1) $$\begin{array}{c} R_{s}\left(S_{i},t\right)=\alpha \;\log\left(S_{i}t\right), \end{array}$$

(2) $$\begin{array}{c} R_{a}\left(A_{k},V_{k}\right)=\sum_{k=1}^{j}A_{k}\log\left(V_{k}\right)S\left(k\right), \end{array}$$

(3) $$\begin{array}{c} R_{c}\left(N_{i}\right)=\gamma_{1}N_{ic}T_{\text{total}}-\gamma_{2}N_{ie}T_{\text{total}}. \end{array}$$

In (1), the *S*_*i*_ denotes the currency amount of the *i*^*th*^ node; the *t* represents the time length that node *i* has owned this currency, *S*_*i*_*t* is the currency age, and *α* is a conversion factor. The PoR consensus mechanism uses the logarithmic formula to calculate reputation value. The reputation value growth rate decreases as the wealth increases; this reduces the gap between the rich and the poor so that people of moderate wealth also have the opportunity to create new blocks for reward of increasing its reputation value.

The *j* in (2) is the number of transactions related to node *i*. With the appropriate settings of the weighting factor *A*_*k*_ and the scaling factor *S(k)*, nodes would prefer to trade with other high reputation nodes to achieve or maintain their high reputation status.

The *R*_*c*_ in (3) incentivize nodes to frequently make positive contributions to consensus voting to increase their reputation values.

The reputation value *R*_*i*_ for each node in the network can be calculated using the following (4) from [9], where *β*_1_, *β*_2_, and *β*_3_ are weighting parameters. Readers are referred to [9] for a more detailed description of each of the parameters in following equations:

(4) $$\begin{array}{c} R_{i}=\beta_{1}R_{s}\left(S_{i},t\right)+\beta_{2}R_{a}\left(A,V\right)+\beta_{3}R_{c}\left(N_{i}\right). \end{array}$$

There is also a positive causal connection between the system currency and the reputation values; the high reputation nodes are likely responsible for the system's security because system security is inseparable from their wealth.

The process of creating a new block is as follows.

1. Select a Leader to create a new block. As shown in Figure 3, an initial reputation ranking block is generated during the system initialization. The highest reputation node of the initial reputation ranking block is selected as the Leader to create blocks 0 and 1. Then, reputation ranking blocks 0 and 1 are built according to the blocks 0 and 1 created by the Leader. The highest reputation node of block 0 creates block 2, the highest reputation node of block 1 creates block 3, and so on. After creating a new block, the Leader needs to sign and broadcast it to the network and wait for the other nodes in the network to vote on it.
2. Votes on the new block. The validation group consists of high reputation nodes, and the sum of their reputation values is over 80% of the system's total reputation values. The nodes in the validation group are usually in the top 20% of the highest reputation nodes. All nodes in the network can verify whether the transactions and signature are legitimate and then vote on it. The Leader needs to collect the voting information and store it in the reputation sub-block as a Merkle tree. The block will be uploaded to the blockchain when (i) more than 2/3 of the validation group nodes vote in favor; (ii) the sum of the YES voters' reputation values exceeds ½ of the system total reputation value. The block is rejected in the opposite scenario.
3. The other nodes in the blockchain network verify the new block. Other nodes verify the newly released block and update their local blockchain data for consistency.

## 3. Redactable Blockchain

We propose a redactable blockchain based on the blockchain structure of PoR, using a new Merkle tree and a one-way trapdoor function. The specific transaction in the *Request* can only be legitimately modified when the nodes who agree to perform the requested modification have more than 1/2 of the whole reputation value in the network, so the amendment represents the system's will. Furthermore, the blocks' link and other data remain unchanged after the amendment. Thus, the proposed redactable blockchain prevents illegal or malicious modifications. We first introduce the redactable blockchain structure and then analyze the modification principle and security.

### 3.1. Structure of Redactable Blockchain

As shown in Figures 4 and 5, the structure of the redactable block uses a new Merkle tree that incorporates the *XOR* operation *H(tx)* on the one-way trapdoor function and the hash function. This operation ensures that the transaction Merkle root, the signature, and the hash value of the block header will remain unchanged after the modification, keeping the links of blocks intact.

The difference between the traditional Merkle tree and the new Merkle tree is in the hashing of the leaf nodes.

In the traditional Merkle tree, the value of each leaf node is the *SHA256* hash *h(tx)* of a transaction *tx*. The parent node's value is the hash of two hash values, *h(tx1)* and *h(tx2),* of the two children nodes, and this hashing process is repeated until the transaction Merkle root is generated. Therefore, we can detect any tamper of transactions according to the Merkle root to ensure the transaction data's integrity [15]. If a transaction is tampered with, its hash value and the transaction Merkle root will also change; therefore, the transactions on the blockchain cannot be modified without being detected at the Merkle root.

In the new Merkle tree structure, the value of the leaf node is *H(tx)*, which is the *XOR* of the hash value *h(tx)* of the transaction *tx* and the one-way trapdoor function *g(x)* (the calculation process of the other nodes remains unchanged):

(5) $$\begin{array}{c} H\left(tx\right)=h\left(tx\right)⊕g\left(x\right). \end{array}$$

*x* is the Leader's exclusive random number, automatically generated when the public and private keys are created and recorded as a common parameter. *g*(*x*) is the result of encrypting the random number *x* with the public key. When the transaction *tx* is modified to *tx*_*new*_, the block Leader can use its private key to compute a new number *x*′ = *g*^−1^, (*h*(*tx*) ⊕ *g*(*x*) ⊕ *h*(*tx*_new_)), to satisfy the formula:

(6) $$\begin{array}{c} h\left(tx\right)⊕g\left(x\right)=h\left(tx_{\text{new}}\right)⊕g\left(x^{\prime }\right). \end{array}$$

Although the transaction is modified, with the calculated number *x*, the transaction Merkle root, the signature, and the other data in the block header remain unchanged; the block header's hash is also intact, therefore maintaining the links of blocks. Thus, the new Merkle tree can still achieve the functions of the traditional Merkle tree as follows:

1. Providing a Merkle proof. *Light nodes* can verify whether a transaction exists by Merkle proof with the help of *full nodes*, even if only the block header is stored (a *full node* has all transactions in the network, while a *light node* only has transactions related to itself).
2. Verifying whether a transaction has been modified. Suppose an attacker wants to change a transaction maliciously. Because only the Leader owns the trapdoor, an attacker cannot calculate the number *x*′ to ensure the transaction Merkle root is unchanged. So, we can judge whether a transaction is modified according to the different transaction Merkle root.

### 3.2. The Principle of Redactable Blockchain

In a redactable blockchain, the data on the blockchain can be legitimately modified in the interest of the system if nodes with more than 1/2 of the system total reputation value agree the modification. Furthermore, the modification does not break the links between the blocks. The following section describes how to implement modification operation and ensure it is legal.

#### 3.2.1. Implementing Data Modification

*(1) Legitimacy Verification of a Modification Request*. When a node has a valid reason to modify a transaction, the node can send a modification *Request* to the network. All nodes in the network could vote on whether the *Request* is legitimate. The *Request* is approved if the sum of the yes voters' reputation values is greater than 1/2 of the system's total reputation value; otherwise, the *Request* is rejected if the voting result is in the opposite. The modification *Request* information includes the height of the block to be modified, the serial number of transactions, the reason of redaction, and the set after redaction.

(7) $$\begin{array}{c} \text{Request}=\left\{{\text{Height,ID,Action,data}}_{\text{new}}\right\}. \end{array}$$

The requirement of high reputation yes voters' sum of reputation values is more than 1/2 of the system's total reputation values ensures the “legality” of the modification *Request*, and prevent malicious nodes in the network from destroying the modification operation. Higher reputation nodes are more likely honest nodes, so these nodes are entrusted with more decision-making power.

*(2) Process of Implementing Data Modification*. The Leader needs to calculate a new number *x*′ = *g*^−1^(*h*(*tx*) ⊕ *g*(*x*) ⊕ *h*(*tx*_new_)), to guarantee that the Merkle root and the data in the block header remain unchanged after the transaction modification. Hence, the links of the blocks are not affected, and there is no need to adjust the data of the subsequent blocks. Furthermore, all nodes in the network can verify the legitimacy of the data at any time.

*(3) Update of System Status*. The Leader generates a new transaction message called *txorg* for traceability after the modification operation is executed. The content of *txorg* is as follows:

(8) $$\begin{array}{c} \text{txorg}=\left\{{\text{id,Height,ID,Action,data}}_{\text{new}},x,x^{\prime },{\text{Pubkey}}_{\text{leader}},\text{time},rt\_\text{set}\right\}. \end{array}$$

The contents of the *txorg*, in sequential order, are as follows:

- The serial number of the *txorg*, *id*
- The height of the block, *Height*
- The serial number of transactions, *ID*
- The reason of redaction, Action
- The set after redaction, datanew
- The Leader's random number, *x*
- The calculated new number, *x*′
- The Leader's public key, *Pubkey*_*leader*_
- The time of modification, *time*
- The voting record to the Request, rt_set

All network nodes can verify the modification's legitimacy according to *txorg* and update their local blockchain data for the consistency of the chain.

Figure 6 illustrates the data modification process.

First, the node sends a transaction modification *Request*.

Second, all nodes send in the network vote on the legitimacy of the *Request*. The *Request* is considered legitimate if the favorable votes come from nodes whose sum of reputation values is more than 1/2 of the system's total reputation values. Then, the Leader executes the legitimate modification *Request* by calculating a new number *x*′ so that the links of blocks are not affected after the modification. Otherwise, reject the modification *Request* and vastly reduce the reputation value of the node sent the *Request*.

Third, the Leader issues a transaction for traceability, and the nodes of the whole network verify whether the executed modification is legitimate and update their local blockchain data.

#### 3.2.2. Ensuring the Legality of Modification

The redactable blockchain does not compromise blockchain security while addressing the limitations of immutability. Because only legal changes voted and verified through by the network's nodes can be performed, the “redactable” blockchain can still ensure the data's security, guaranteed by the characteristics of the one-way trapdoor function and our scheme.

We can only adjust the number *x*′ to match the modification of transactions, which guarantees that data and the links of the blocks remain unchanged after the modification. The property of the one-way trapdoor function determines that only the node knowing the trapdoor can find the only number *x*′ that can match the transaction change to execute the modification. In this paper, the trapdoor is the Leader's private key, so only the Leader can calculate the new number, and only the Leader can execute the modification authorized by the network.

Specifically, we choose the SM2 asymmetric cryptography algorithm as the one-way trapdoor function. In essence, the Leader encrypts its selected random number *x* with its *public key*. According to the one-way trapdoor function properties, all nodes can use the Leader's *public key* to calculate *g(x)* given *x*. However, only the Leader can do the reverse calculation, that is, calculate *x* given *g(x)*, with the corresponding *private key*. Therefore, the Leader's private key is the trapdoor generated by one-way trapdoor function. Furthermore, the blockchain modification request needs to be approved by the nodes in the network before execution and verified by all other nodes after implementation. Therefore, the modification operation represents the will of the system and is legitimate.

#### 3.2.3. Security Analysis of Data Modification

To illustrate the security of the redactable blockchain scheme, we simulate the attacks of a malicious adversary on modifying block transactions. The adversary can take the following methods:

1. Modify the target block data, modify the data of all blocks on the chain from the targeted block up to the latest block, and keep the links of blocks unchanged
2. Calculate a new number for the modification so that the new Merkel tree root is unchanged after modifying the targeted block data

Attack scenario 1 is not feasible because only the block Leader can modify the block. Furthermore, the Leader of each block on the path from the targeted block up to the latest block may be different. The Leaders of each block on the block path are all high reputation nodes. A high reputation node is likely trustworthy because its wealth is closely related to the system's security. According to the principle of maximum wealth, high reputation nodes will not damage the system, negatively affecting their wealth. So, the adversary cannot perform all modification operations from the targeted block up to the latest block. Therefore, the adversary's attack is not feasible.

The attack scenario 2 is also infeasible because only the Leader knows the trapdoor of the new Merkel tree, so only the Leader can calculate the unique number to keep the Merkel root unchanged after the transaction modification. And the Leader with a high reputation is more likely to be honest because blockchain security is closely related to its wealth. However, suppose the Leader does not faithfully execute the modification request in the network. In that case, the unauthorized modification cannot pass the verification of the other nodes, and the modification operation cannot complete. The Leader's reputation value is also significantly reduced as a consequence. In this way, the attacker cannot obtain benefits but loses his wealth, violating the principle of attack. Therefore, the scheme is safe. In conclusion, the redactable blockchain scheme is safe and effective.

## 4. Experimental Simulation

Smart contracts can be used for computing devices management in MEC. However, if a smart contract with bugs is released in MEC, and the bugs can cause devices to fail to alert potential warning conditions, it can cause irreparable damage. In this scenario, the proposed redactable blockchain scheme can modify the uploaded buggy smart contract to prevent damage that the buggy smart contract can cause. For easier understanding, the information in the buggy smart contract can be treated as transaction data in the system blockchain to implement the modification. Furthermore, the proposed redactable blockchain also facilitates companies' compliance to GDPR, the EU law on data protection and privacy. For example, in a blockchain-based electronic health record system, the medical institute should ensure that customer's personal data are accurate and up to date, and be able to modify customers' personal data or completely erase a customer's health record at the customers' request. In these scenarios, the customers' health records can be treated as transaction data modified or deleted.

We simulated the data modification on a blockchain under the PoR consensus mechanism. The experiment uses Python as the language, PyCharm, as the compiler and imports the encrypted package of gmssl.sm2 for the encryption, decryption, and signature operations.

### 4.1. Competition of Bookkeeping Rights

Table 1 shows the information of the nodes in the initial system. There are no transactions and validation votes in the initial system, so the reputation values are only related to the nodes' wealth.

The system converts the amount of currency into a reputation value using the conversion formula in equation (1), that is, *R*_*s*_(*S*_*i*_, *t*)=*α*  log(*S*_*i*_*t*), and generates an initial ranking of reputation value, as shown in Table 2. We set the conversion factor *α* as 1/2. The initial reputation value is only related to currency amount because no transactions have been generated yet.

Figure 7 shows the nodes' reputation values.

The consensus mechanism selects the highest reputation node as the Leader to create a new block. Then, other nodes in the network vote on the legitimacy of the new block, and all nodes can verify the legitimacy of the new block.

### 4.2. Generation of New Blocks

The system sets each block to pack four transactions. The initial reputation ranking determines that node 1 is the Leader to create blocks 0 and 1. The Leader collects four transactions in the transaction pool, packs them into a block, and releases it to the network with a signature. All nodes in the network vote on the legitimacy of the transaction and verify the signature. If passing the validation, the block is uploaded as block 0, and a new reputation ranking table 0 is generated. The highest reputation node in reputation ranking table 0 generates block 2. Similarly, the highest reputation node in reputation ranking Table 1 generates block 3, and so on.  Figure 8 shows the detailed structure of blocks 0 and 1.

Let's use block 1 as an example to introduce the computation of the transaction Merkle root.

1. Block 1 contains four transactions, and node 1 is the Leader of block 1. The one-way trapdoor function *g(x)* can be calculated using SM2 encryption on the Leader's exclusive random number *x* using the public key of the Leader (node 1). The *g(x)* is at least 776 bits in length. We calculate the *SHA256(tx)* of each transaction first and then pass the value of *SHA256(tx)*^*∗*^*3* to the first 768 bits of *h(tx)*, and padding the remaining bits of *h(tx)* with zero to make *h(tx)* and *g(x)* equal in length. Then, calculate the hash value *H(tx)* of each leaf node.
2. After calculating the *H(tx*_*i*_) of each Merkle tree leaf node *i*, we compute the hash value of the parent node of two leaf nodes by performing *SHA256()* hashing of the concatenation of their hash values. These steps are repeated until the transaction Merkle root is generated.

(9) $$\begin{array}{c} \text{Merkle root}=\text{SHA}256\left(SHA256\left(H\left(tx1\right)\left\|H\left(tx2\right)\right)\right)\left\|\text{SHA}256\right)\left(Ht\left(x3\right)\left\|H\left(tx4\right)\right)\right)\right). \end{array}$$

The value of *g*(*x*) is as follows:

(10) $$\begin{array}{c} g\left(x\right)=\text{efcd}19\text{ddc}10422480\text{f}18792\text{b}6\text{d}77\text{be}29\text{f}288\text{f}644\text{cb}4\text{b}1625\text{c}9754\text{f}7\text{aa}00\text{c}8\text{f}93304\text{df}99\text{bcf}6188\text{b}139\text{e}429\text{d}07\text{d}78\text{d}8177\text{a}90\text{babaec}7\text{e}7\text{b}7\text{b}42\text{b}6\text{bcb0ed}6\text{e}9712\text{e}9\text{c}986111\text{fda}10\text{b}602\text{d}99\text{f}4\text{a0d}64\text{f}2\text{e}9\text{a}566324432\text{d}8990810412\text{e}3\text{d}215\text{f}0083\text{a}5\text{df}14\text{ec.} \end{array}$$

Table 3 shows the hash of transactions.

We can calculate the Merkle root according to Figure 9:

(11) $$\begin{array}{c} \text{Merkle root}:3d8430dc65c27e587633600426c43\text{feea}1b9\text{eae}232063ea11001fcb88ff513ec. \end{array}$$

The private key of block Leader (node 1) is as follows:

(12) $$\begin{array}{c} \text{private\_key}:2\text{b}40\text{bbd}922\text{b}8\text{cb}4\text{f}99\text{a}67875\text{b}35440562133\text{d}7\text{cf}6\text{ac}9710\text{a}60\text{d0baaefdca}6\text{b}54\text{.} \end{array}$$

The signature of the block Leader (node 1) to the block header is as follows:

(13) $$\begin{array}{c} \text{Sign}:94532\text{e}3\text{d}3\text{d}8\text{afa}58838\text{c}4\text{f}5\text{c}2137\text{fa}3\text{c}3\text{dc}7\text{e}4\text{eaf}290\text{b}1\text{d}2595\text{e}2\text{ad}633\text{e}7\text{d}13\text{e}\\ 7\text{aeae}4656\text{ff}1\text{d}317952245\text{b}795\text{cff}894316\text{e}9\text{bad}0714\text{be}778569\text{be}9225\text{e}525\text{e}9\text{.} \end{array}$$

The block Leader (node 1) publishes the packaged block and signature to the network. Then, all nodes in the network vote on the legitimacy of the transactions and verify the signature in the block. Next, the block Leader (node 1) collects the vote information and stores it in the reputation sub-block. After the nodes finish the validation and vote in agreement for the block, block 1 is officially uploaded. After block 1 Leader (node 1) uploads block 1, the rest nodes in the network verify the legitimacy of block 1 and update their local blockchain data to achieve the consistency of the distributed data if passing the verification.

### 4.3. Modification of Block Data

Suppose a blockchain-based health record system needs to update a customer's personal data in compliance with GDPR at the customer's request. Under the EU General Data Protection Regulation (GDPR), Bob as a customer is entitled to demand his personal data be accurate, be up to date, or be deleted. For example, Bob can request that his contact information be updated after he has changed a phone number or moved to a new address. For example, Bob informs his hospital that he has moved home. His hospital is obliged to update Bob's personal information, and the hospital can send an “Address change” *Request* to the medical blockchain system with Bob's ID.

(14) $$\begin{array}{c} \text{Request}=\left\{{}^{\prime }\text{Height: }0^{\prime }\text{,}{}^{\prime }I\;D\text{ : }2^{\prime }\text{,}{}^{\prime }\text{Action}:\text{customer changed address,Address :}78\text{ some street,zheng zhou}\right\}. \end{array}$$

All nodes (participating hospitals) in the blockchain-based health record system validate whether the modification request is legitimate. If they approve the modification request, the Leader of block 1 performs the modification as shown in Figure 10 to update this customer's personal record. Block 1 Leader (node 1) can calculate a new number *x*′ to execute the amendment without affecting the transaction Merkle root and the links of blocks.

The new number *x*′  = g-1 (*h*(*tx*) ⊕ *g*(*x*) ⊕ *h*(txnew)) is calculated, which satisfies (6).

The hash of *tx2*_*new*_ is as follows:

(15) $$\begin{array}{c} SHA256\left(tx2_{\text{new}}\right)=\;5\text{f}03\text{ca}15\text{f}22\text{bf}2\text{faebea}168783\text{fdb}976\text{a}740\text{e}00744\text{eb}9\text{b}7\text{b}7240\text{b}6586\text{b}8\text{b}1269\text{.} \end{array}$$

The value of *g(x′)* is as follows:

(16) $$\begin{array}{c} g\left(x^{\prime }\right)=7\text{a}9299\text{a}80\text{e}5\text{a}161\text{b}37\text{de}114\text{f}81\text{c}5\text{f}959211\text{c}65\text{b}1\text{e}8\text{c}0599\text{e}26507593\text{bed}1087\text{aa}51279\text{ee}003\text{fbce}2012241\text{b}491\text{ca}9\text{f}67\text{a}90\\ 4294\text{fcff}534\text{c0ad}938659\text{f}3\text{b}310\text{fb}7\text{c}960664\text{d}08424\text{e}53\text{a}1\text{ff}72\text{ee}1\text{d}6\text{b}59976\text{f}2\text{a}1\text{b}11153\text{d}6\text{b}3\text{ff}6414\text{d}43\text{f}82876\text{aa}5\text{df}14\text{ec.} \end{array}$$

Decryption to calculate the new number is as follows:

(17) $$\begin{array}{c} x^{\prime }=1183451931\left(468a0b1b\right). \end{array}$$

Figure 11 shows the result of the program. We can calculate the result of *XOR* operation. Therefore, the transaction Merkle root is the same after updating this customer's health record.

The signature and the hash of the block header will not change if the transaction Merkle root does not change after the modification, so the links of blocks are not affected. After completing the modification, block 1 Leader (node 1) generates a new transaction record called *txorg* and publishes it to the network, as shown in Figure 12, for legitimacy verification by the rest nodes in the network.

The other nodes in the network verify whether the modification is legal according to *txorg*, and update their local blockchain data if the amendment is legitimate, which completes the modification operation.

After the modification, both the transaction Merkle root and the block header's hash are unchanged; the links of blocks are not affected, so the modification operation is feasible.

## 5. Conclusion

A redactable blockchain scheme based on the PoR consensus mechanism is put forward in this paper to address the problem of amending or removing erroneous or sensitive data on blockchains of MEC applications. The proposed Merkel tree structure uses the one-way trapdoor function characteristics, which ensures the Merkle root does not change after modifying a transaction, so the links of blocks are not affected. Although only the block Leader node with the trapdoor can legally perform the modification operation, the modification operation also needs to be validated and agreed upon by the nodes of the whole network to ensure the integrity and security of the blockchain.

## Figures and Tables

**Figure 1:** Block structure [9].

**Figure 2:** Details of a vote information.

**Figure 3:** Process of creating new blocks [9].

**Figure 4:** Structure of redactable block.

**Figure 5:** Traditional Merkle tree and new Merkle tree.

**Figure 6:** Process of data modification.

**Figure 7:** Nodes' reputation values.

**Figure 8:** Blocks 0 and 1.

**Figure 9:** Computation of the Merkle root.

**Figure 10:** Operation of the Leader.

**Figure 11:** Program result.

**Figure 12:** Details of transaction record *txorg.*

**Table 1:** Node information.

Id	Public key	Wealth	Random number
1	87979b12e898279dfae24641faf44b10b9c623484224e5b0b8929731e31276af 41d3d810d04038fece131e38c28106429bbfe325d6bc0f9a46f34a8b2b0f4a82	10000	635635635
2	e9f783b762a864afb2b2483a8d92f4a0f979fd49b89506092b6b7cdc7fb1bba9 14fd193514171f9eeb480424275fde4bb8d1e895f4afb315f012137135d33ed0	6000	359147852
3	de31612374ea9e9a8f7e7d2d6650f32bdcc780f2749f4edb25f9e09d7726f8bf 2a623e2fbf708dfaee87c68abdd5072c830cc350832f8cace015f57b8897f887	3000	972951361
4	e88f5ce03fa86f77b19f42d59c59e1a69f4ab714ba9006f50255165a530be1d5 4a9899009bcb895636c90079f92938b902ffb4f570a80859e585f2668fdc1087	8000	168752164
5	83f6eb2bbd6265db7f6ef738ccb294d5078c64071804e6b81863f049bf5b630c aefa0918f850449eb37bd16796b4e3295f969f0e1306952374dcfa9011bd50f3	500	160789451
6	d36906b0d14e4280b2a74ec925a574f1d632378b8a2efd25ac30f17c02c6d2b7 93a888cd3c8253fa216bba67e8324c8e3de5da8d9e3abc3bfed9b4bde6ea074	800	938852164
7	8ab479c2bd550973e773f336ca94612bfa404723ddc0000f6d76eae32d2f8278 7484dec28e603f3b6a9f8ec01509c0a742a4de7ffe467c4c62e091dd124a4f15	2000	543163456
8	7d36518d966e5015274c7a78c19620b71e0771838c0e779eb5ca2bd070bd819 51a8030f0a455e2c7b752ac35c885f3f41d3f36c1d8c1ba8b4860dc312bca659	100	700785426
9	61388661dd35fdf73b8da16f9c49d6420ce780c95fa0a6fb7ef73ac3d87debb15 ca44be28820e3b113641c8351c759a6bd73f5d598b724e5367611f23dfc11d0	0	844111594
10	98dd03004e355417668d8ea016085e8dd64a2f788ea95052b1a2058ca8ea81cf 3366f883b4279762414b5e68c7f9fd35c27ccbc1174df00fb222ec0b83f557c0	50	162111021

**Table 2:** Ranking of initial reputation.

Id	Wealth	Reputation value
1	10000	8.30482023
4	8000	8.14385619
2	6000	7.93633744
3	3000	7.43633744
7	2000	7.14385619
6	800	6.48289214
5	500	6.14385619
8	100	4.98289214
10	50	4.48289214
9	0	0

**Table 3:** Hash of transactions.

Transaction	SHA256()
*tx1*	70d78a190451aaeadfbccc0ddf1043c7a6851595dcc01cb13a1953df57e9cbee
*tx2*	ca5c4a603d75c6a9d32c7ee36f4ffe0674d473f26760d4c09d658cb175569580
*tx3*	6de64c719e4d7604af8c3120ecdfc559217a68246389b4ba4422fbc6c381d924
*tx4*	8586e0ec5a2f382394cc04d57f1b032cb22b94927f468d2c21b142f227b27f35

## Data Availability

Our experimental results are available from the corresponding author upon request.

## References

[1] Guo S., Dai Y., Guo S., Qiu X. F. (2020). Blockchain meets edge computing: stackelberg game and double auction based task offloading for mobile blockchain. *IEEE Transactions on Vehicular Technology*.

[2] Qu Z., Sun H., Zheng M. (2021). An efficient quantum image steganography protocol based on improved EMD algorithm. *Quantum Information Processing*.

[3] Zhaofeng M., Xiaochang W., Jain D. K., Khan H. G. W. (2020). A blockchain-based trusted data management scheme in edge computing. *IEEE Transactions on Industrial Informatics*.

[4] Yuan Y., Wang F.-Y. (2018). Blockchain and cryptocurrencies: model, techniques, and applications. *IEEE Transactions on Systems, Man, and Cybernetics: Systems*.

[5] Zaghloul E., Li T., Mutka M. W., Ren J. (2020). Bitcoin and blockchain: security and privacy. *IEEE Internet of Things Journal*.

[6] Tomić N. Z. (2021). A Review of consensus protocols in permissioned blockchains. *Journal of Computer Science Research*.

[7] Xiao Y., Zhang N., Lou W., Hou Y. T. (2020). A survey of distributed consensus protocols for blockchain networks. *IEEE Communications Surveys & Tutorials*.

[8] Qu Z., Huang Y., Zheng M. (2020). A novel coherence-based quantum steganalysis protocol. *Quantum Information Processing*.

[9] Zhuang Q. W., Liu Y., Chen L. S., Ai Z. Proof of Reputation: A Reputation-Based Consensus Protocol for Blockchain Based Systems.

[10] Huang K., Zhang X., Mu Y. (2019). Building redactable consortium blockchain for industrial internet-of-things. *IEEE Transactions on Industrial Informatics*.

[11] Li c., Rao H., Xu A., Guo X. H. (2018). Strategic research on China energy technology revolution system. *Chinese Journal of Engineering Science*.

[12] Ren Y. L., Xu D. T., Zhang X. P., Eng X., Wu G. D. (2020). Scheme of revisable blockchain. *Journal of Software*.

[13] Politou E., Casino F., Alepis E., Patsakis C. (2021). Blockchain mutability: challenges and proposed solutions. *IEEE Transactions on Emerging Topics in Computing*.

[14] Qu Z., Chen S., Wang X. (2020). A secure controlled quantum image steganography algorithm. *Quantum Information Processing*.

[15] Lee D., Park N. (2021). Blockchain based privacy preserving multimedia intelligent video surveillance using secure Merkle tree. *Multimedia Tools and Applications*.

